This article has been retracted.

# The Change of Soluble Programmed Death Ligand 1 (sPD-L1) in Plasma of Small Cell Lung Cancer and Its Clinical Significance

**DOI:** 10.1155/2022/8375349

**Published:** 2022-01-28

**Authors:** Feijie Lu, Yongquan Dong, Qianjun Li, Mingming Wang

**Affiliations:** Department of Respiratory Disease, Yinzhou No. 2 Hospital, Ningbo, Zhejiang Province, China 315040

## Abstract

Background soluble programmed death-ligand 1 (sPD-L1) expression in lung squamous cell carcinoma and lung adenocarcinoma is associated with disease progression, and sPD-L1 expression in small cell lung cancer (SCLC) may have similar manifestations and become a potential marker for treatment. The purpose of this study was to observe the changes of plasma sPD-L1 expression in SCLC patients. *Methods*. 90 patients diagnosed with SCLC from January 2019 to November 2020 were selected as the test group, including 72 males and 18 women, 58.7 ± 6.6 years; 30 healthy subjects were selected from the physical examination center, including 18 males, 12 females, and 60.3 ± 7.0 years. There were no statistical difference in sex and age factors between the trial and control groups (*p* > 0.05). Selected SCLC used chemotherapy regimen: cisplatin + etoposide (EP), carboplatin + etoposide (CE), and SCLC group were divided into three subgroups of disease progression group, partial remission group, and disease stability group according to the treatment effect. Comparison of the differences in sPD-L1 expression content between the experimental and control populations. Plasma sPD-L1 levels were dynamically monitored pre- and posttreatment in 90 patients with small-cell lung cancer and were associated with efficacy among subgroups. Meanwhile, the risk factors for patient sPD-L1 expression content were analyzed by logistic regression. *Results*. Plasma sPD-L1 levels were higher in the SCLC group than in the healthy people group (*t* = 7.40, *p* < 0.01). In the disease progression group of the SCLC group, sPD-L1 levels were decreased in the SCLC group, sPD-L1 in some remission group was increased after treatment, and sPD-L1 levels in the disease-stable group (*p* > 0.05). Multivariate logistic regression analysis showed that factors promoting increased sPD-L1 expression in SCLC patients included increased smoking, brain metastasis, and ProGRP expression (both *p* values < 0.05). *Conclusion*. (1) Higher peripheral sPD-L1 expression in SCLC patients than in healthy patients, and the expression levels were closely related to efficacy. (2) Dynamic changes in s PD-L1 were correlated with clinical efficacy. (3) The progression of sPD-L1 and ProGRP in SCLC patients showed the same extent during remission and stabilization, suggesting the effect of s PD-L1 in the evaluation of SCLC tumors and the reflection of the tumor marker ProGRP.

## 1. Introduction

The annual incidence and mortality rate of lung cancer are the first in the world, and lung cancer is also the primary cause of death of cancer in China [1, 2]. Lung cancer is divided into two main histological types: nonsmall-cell lung cancer (NSCLC) and small-cell lung cancer (SCLC). SCLC accounts for about 15% of the total lung cancer, with the highest degree of malignancy and mostly occurs in the middle of the lung, and it grows rapidly, has early metastasis, and has a neuroendocrine function [3]. The tumor marker gastrin-releasing peptide precursor (ProGRP) is a potent tumor marker in early SCLC and can be significantly elevated in the serum of restricted SCLC patients with high sensitivity and high specificity [4].

Promed death 1 receptor (PD-1) is a receptor protein present on the surface of immune cell T cells acting with programmed death-ligand 1 (PD-L1), and PD-L1 is a protein expressed on the surface of tumor cells [5]. It has been shown that the expression of PD-1/PD-L1 binding is abnormally elevated in tumor tissue and may play an important role in tumorigenesis and development [5]. The combination of PD-1 and PD-L1 transmits negative regulatory signals to T cells to induce T cells into a dormant state; T cell proliferation decreases, resulting in being unable to identify and kill tumor cells, thus, making tumor cells more likely to proliferate and metastasis [6]. And recent studies have shown that multiple immunotherapy trials on blocking the PD-1/PD-L1 pathway in SCLC have achieved better results compared to conventional chemotherapy.

PD-L1 is divided into two types: membrane-type (mPD-L1) and soluble (sPD-L1). Domestic studies have found that peripheral blood changes in sPD-L1 were associated with disease progression in patients with lung cancer before and after chemotherapy, but this study only included patients with lung squamous carcinoma and lung adenocarcinoma, and the changes in SCLC patients have not been fully studied [7]. This study was designed to evaluate the expression level of sPD-L1 in SCLC patients, to analyze its changing trends in different efficacy, and to analyze its correlation with ProGRP.

## 2. Data and Methods

### 2.1. Diagnostic Criteria for the SCLC

Diagnostic criteria for SCLC refer to the <Individualized Treatment of Lung Cancer> [8]: the diagnosis of SCLC is mainly comprehensively judged by medical history, physical examination, hematological examination, imaging examination, endoscopic examination, and pathological examination. (1) The first symptoms of clinical diagnosis include cough, sputum, fever, chest tightness, shortness of breath, chest pain, and extrapulmonary symptoms, especially for middle-aged and elderly men who smoke for a long-term time; they should undergo chest CT examination in time. (2) Imaging diagnosis of chest CT has become the preferred examination method to diagnose small cell lung cancer. CT combined with percutaneous lung puncture biopsy, fiber bronchoscopy biopsy, and other methods can significantly improve the diagnosis rate of small cell lung cancer.

### 2.2. Inclusion and Exclusion Criteria

Inclusion criteria for this study: (1) meet the patients diagnosed with SCLC; (2) first diagnosed in the hospital, not treated; (3) informed of their own condition; and (4) agree to accept the experiment and sign the study consent form. Exclusion criteria for this study: (1) psychiatric patients or other patients who cannot cooperate; (2) incomplete medical records or replaced other treatment methods or hospital patients; (3) severe internal cerebral organic or vascular lesions, liver, and kidney metabolic dysfunction; and (4) patients without interrupted treatment or withdrawal for various reasons.

### 2.3. General Patient Data

Small cell lung cancer group: after screening with the above criteria, 90 naive patients diagnosed with SCLC by pathological examination from January 2019 to November 2020 were included in the trial group, including 72 men and 18 women, aged 58.7 ± 6.6 years. The selected patients had complete medical records, including gender, age, smoking status, and tumor stage (see Figure 1 for the screening process). Healthy control group: 30 patients were selected from the physical examination center as the control group, including 18 men and 12 women, aged 60.3 ± 7.0 years old. There were no statistical differences between gender, age, and other basic information and the test group (*p* > 0.05). General data of the two groups are shown in Table 1.

### 2.4. Collection of Specimens

In this assay, 3 ml of peripheral blood from the SCLC and healthy groups was collected and placed in EDTA anticoagulant tubes, centrifuged at 2000 g within 30 min for 5 min, upper plasma was absorbed by disposable suction tubes, and the same specimens were placed in 2 EP tubes for numbering and preservation. Plasma levels of sPD-L1 expression were measured in healthy subjects by the ELISA method, according to the kit instructions and operating specifications.

### 2.5. Treatment Methods and Observation Indicators

SCLC patients use the chemotherapy regimen: cisplatin + etoposide (EP) and carboplatin + etoposide (CE) systemic chemotherapy for 4 cycles, to evaluate the treatment effect. The efficacy of SCLC patients was evaluated according to the evaluation criteria of the 2016 edition of the <Individualized Treatment of Lung Cancer> [8] and was divided into disease progression, partial remission, and disease stable groups. Peripheral blood was harvested for 3 mL/time during partial chemotherapy, centrifuged at 2 000 r/min for 10 min within 30 min, and the primary supernatant was taken and kept at-70°C. The expression levels of sPD-L1 and ProGRP were determined by the ELISA assay.

### 2.6. Statistical Method

Data analysis was performed using SPSS21.0 statistical software. Measurement data are indicated as (*x* ± *s*), group comparison using independent sample *t*-test; count data by [*n* (%)], group comparison by 2 test, *p* < 0.05 is statistically significant. Univariate logistic regression analysis was used to screen for independent variables that were potentially dangerous for sPD-L1, where factors for *p* 0.10 and clinically important indicators were included in the multivariate logistic regression equation to analyze independent risk factors for sPD-L1.

## 3. Result

### 3.1. The Levels of sPD-L1 Expression Were Observed in Both Groups

Peripheral sPD-L1 levels in lung cancer were (1.74 ± 0.82) ng/ml and (0.59 ± 0.33) ng/ml, and sPD-L1 in lung cancer than benign and controls (*p* < 0.01) is shown in Table 2.

### 3.2. Changes in sPD-L1 Levels in the Peripheral Blood during the Treatment

SCLC patients received systemic chemotherapy to compare changes in sPD-L1 levels during chemotherapy in the disease progression, partial remission, and disease stable group. The *p* values were < 0.01 in both the disease progression and partial remission groups, indicating a statistically significant mean difference in sPD-L1 content between the disease progression and partial remission group, see Figure 2.

### 3.3. Changes in ProGRP Levels in Peripheral Blood before and after Treatment

SCLC patients compared changes in chemotherapy course ProGRP levels in disease progression, partial remission, and disease stable groups before and after receiving systemic chemotherapy. The *p* values were < 0.01 in both the disease progression and partial remission groups, indicating that the mean difference of ProGRP content was significant before and after chemotherapy, see Figure 3.

### 3.4. Logistic Regression Analysis of the Clinical Characteristics of sPD-L1 with SCLC Patients

The results of the univariate Logistic regression analysis showed that the tumor stage, stage, smoking, brain metastasis, and the increased ProGRP expression content were the influencing factors of the increased sPD-L1 expression. After adjusting for other factors, the results of the multivariate logistic regression analysis showed that the factors promoting increased sPD-L1 expression in SCLL patients included increased smoking, brain metastasis and ProGRP expression content (both *p* values < 0.05), see Table 3.

## 4. Discussion

In this study, sPD-L1 levels were significantly higher in the SCLC group compared with the control group, suggesting high sPD-L1 expression in SCLL patients. The sPD-L1 levels were decreased in the disease progression group, sPD-L1 in the partial remission group, and relatively small fluctuations of sPD-L1 in the disease-stable group. The reason for the different changes in sPD-L1 content on chemotherapy may be that the level of sPD-L1 expression in vivo is proportional to the inhibitory effect on T cells, and the inactivated T cells after inhibition cannot remove tumor cells, making them escape immune surveillance and thus easier tissue infiltration and distant metastasis [9]. Related studies found that sPD-L1 expression was closely related to the stage of tumor progression and tumor organ metastasis [10]. In this study, sPD-L1 expression in the SCLL group was associated with history of smoking, brain metastasis, and ProGRP expression content. This complements the evidence from previous studies.

Small cell lung cancer has the characteristics of high malignancy, strong invasion, and easy metastasis and mainly relies on chemiotherapy and chemotherapy. PD-1/PD-L1 pathway block inhibitors have become a new breakthrough point in the treatment of SCLC in nearly 20 years. Previous studies have found that plasma sPD-L1 has high specificity and sensitivity in reflecting SCLC tumors and may become a novel SCLC tumor marker [11]. In this study, the sPD-L1 levels were significantly higher in the SCLC group compared with the controls, consistent with previous studies. However, another result of the present study showed that the mean difference of ProGRP content was significantly between the two groups before and after chemotherapy, and logistic regression analysis showed that increased ProGRP content was an influencing factor of increased sPD-L1 expression, and that sPD-L1 and ProGRP changed to the same extent during progression, remission, and stability in SCLC patients. ProGRP is a specific tumor marker of SCLC, which has more advantages over other tumor markers in terms of tumor specificity, release volume, and organ specificity [12]. Moreover, the concentration of ProGRP in the blood is less affected by activity, diet, and other factors, with little daytime fluctuation, and hemolysis has little impact on its test results, so ProGRP facilitates the monitoring of SCLC patients under treatment and contributes to the detection of recurrent cases [13, 14]. Combined with the results of this study, it can be speculated that the effect of sPD-L1 in the assessment of SCLC tumorigenesis and the reflection of the tumor marker ProGRP are close.

Similarly, the present findings found that the factors that promoted increased sPD-L1 expression in SCLC patients also included smoking and brain metastases. Previous studies have shown that smoking is one of the important risk factors for the progression of SCLC [15, 16]. Brain metastasis of lung cancer is a serious complication of advanced lung cancer patients [17]. It can be speculated from this study that smoking-induced SCLC may be associated with smoking promoting sPD-L1 expression, and sPD-L1 may also be one of the markers of metastasis in patients with SCLC. Previous studies have reached the same conclusion by examining the expression of sPD-L1 in tissue samples [18]. However, tissue sample testing has other factors, such as the inconsistent clinical prediction effect, the inability to balance the tumor heterogeneity, the influence of treatment and other intervention factors, the poor detection reproducibility, and the difficulty to simultaneously detect the expression of tumor cells and tumor-infiltrating immune cells. PD-L1 immunohistochemical detection in tissue is difficult to be a predictive indicator of the best dynamic observation for people who benefit from accurately choosing immunotherapy. Compared with tissue specimens, plasma testing can homogenize tumor heterogeneity through plasma testing, more objectively reflect the actual situation of the tumor, is relatively simple in clinical use, and can dynamically and continuously observe changes in indicators. With the widespread application of PD-1/PD-L1 pathway block inhibition in clinical practice, the need for screening accurate and observable biomarkers is even more urgent, and the potential application value of sPD-L1 has gradually been concerned.

## 5. Limitation

One of the limitations of this study lies in the collection of cases and the statistics of the data, where the influence of various influencing factors on sPD-L1 expression should be further analyzed from multiple angles. Although a certain number of data statistics were conducted in this trial, the statistical samples are still small, and a large number of randomized controlled studies are still necessary in the future. Therefore, in the future experimental research, the collection of the study sample size should be increased, and the interaction between the influencing factors should be compared and analyzed, and extend the follow-up time as long as possible to draw a more comprehensive conclusion and better guide the treatment of SCLC patients.

## 6. Conclusion

1. Peripheral blood sPD-L1 expression was higher in SCLC patients than in healthy individuals, and the expression levels were closely related with efficacy
2. Dynamic changes in sPD-L1 were correlated with clinical efficacy
3. The progression of sPD-L1 and ProGRP in SCLC patients showed the same extent during remission and stabilization, suggesting the effect of sPD-L1 in the evaluation of SCLC tumors and the reflection of the tumor marker ProGRP

## Figures and Tables

**Figure 1:** Experimental participant screening process.

**Figure 2:** Changes in sPD-L1 levels in the peripheral blood during the treatment.

**Figure 3:** Changes in ProGRP levels in the peripheral blood before and after treatment.

**Table 1:** General information for two groups of patients $\left(\bar{x}\pm s\right)$.

Characteristics	Experimental group (*n* = 90)	Control group (*n* = 30)
Sex (male/female)	72/18	18/12
Age (age)	58.7 ± 6.6	60.3 ± 7.0
Number of smokers (example)	57	14
Tumor stage (example)		
I stage	8	—
II stage	8	—
III stage	31	—
IV stage	43	—

**Table 2:** Comparison of sPD-L1 expression levels between the two patient groups (*x* ± *s*).

Group	sPD-L1 expression levels (ng/ml)
Experimental group (*n* = 90)	1.74 ± 0.82
Control group (*n* = 30)	0.59 ± 0.33
*t*	7.40
*p*	<0.01

**Table 3:** Logistic regression analysis of clinical characteristics of sPD-L1 and SCLC patients.

Variable	Univariate logistic analysis			Multivariate logistic analysis		
	OR	95% CI	*p* value	OR	95% CI	*p* value
Female	0.62	0.27~0.81	0.35	0.51	0.22~1.02	0.13
Age (per 1 year increase)	1.056	0.75~1.05	0.76	1.04	0.93~1.07	0.57
Tumor staging						
Phase I	2.08	0.88~8.03	0.54	1.37	0.89~1.62	0.58
Phase II	1.06	0.47~2.45	0.04	1.22	0.30~4.83	0.47
Phase III	1.53	0.82~3.66	0.08	1.70	0.64~5.08	0.32
Smoking history (years)	2.56	1.30~6.06	0.01	2.74	0.9I~7.04	0.04
Lung cancer brain metastasis (case)	1.95	0.97~0.99	0.01	1.27	0.94~0.98	0.01
Lung cancer liver metastasis (case)	1.05	0.81~0.99	0.63	0.97	0.84~1.12	0.44
ProGRP (per 1 ng/mL increase)	2.04	1.84~3.99	0.01	1.50	1.04~2.86	0.01

## Data Availability

Data are contained within the article or are available from the individual studies that were referenced throughout the text.
